The article "Angiotensin-converting enzyme 2/angiotensin-(1–7)/Mas axis prevents lipopolysaccharide–induced apoptosis of pulmonary microvascular endothelial cells by inhibiting JNK/NF–κB pathways" was retracted in 2026. Reasons: plagiarized images; duplicated images; overlap with other authors' work; overlap with earlier publications.

# Angiotensin-converting enzyme 2/angiotensin-(1–7)/Mas axis prevents lipopolysaccharide–induced apoptosis of pulmonary microvascular endothelial cells by inhibiting JNK/NF–κB pathways

**DOI:** 10.1038/srep08209

**Published:** 2015-02-03

**Authors:** Yingchuan Li, Yongmei Cao, Zhen Zeng, Mengfan Liang, Ying Xue, Caihua Xi, Ming Zhou, Wei Jiang

**Affiliations:** 1 Department of Anesthesiology, the Sixth People's Hospital Affiliated to Shanghai Jiaotong University, Shanghai 200233, China

## Abstract

ACE2 and Ang–(1–7) have important roles in preventing acute lung injury. However, it is not clear whether upregulation of the ACE2/Ang–(1–7)/Mas axis prevents LPS–induced injury in pulmonary microvascular endothelial cells (PMVECs) by inhibiting the MAPKs/NF–κB pathways. Primary cultured rat PMVECs were transduced with lentiviral–borne *Ace2* or shRNA–*Ace2*, and then treated or not with Mas receptor blocker (A779) before exposure to LPS. LPS stimulation resulted in the higher levels of AngII, Ang–(1–7), cytokine secretion, and apoptosis rates, and the lower ACE2/ACE ratio. *Ace2* reversed the ACE2/ACE imbalance and increased Ang–(1–7) levels, thus reducing LPS–induced apoptosis and inflammation, while inhibition of *Ace2* reversed all these effects. A779 abolished these protective effects of *Ace2*. LPS treatment was associated with activation of the ERK, p38, JNK, and NF–κB pathways, which were aggravated by A779. Pretreatment with A779 prevented the *Ace2*–induced blockade of p38, JNK, and NF–κB phosphorylation. However, only JNK inhibitor markedly reduced apoptosis and cytokine secretion in PMVECs with *Ace2* deletion and A779 pretreatment. These results suggest that the ACE2/Ang–(1–7)/Mas axis has a crucial role in preventing LPS–induced apoptosis and inflammation of PMVECs, by inhibiting the JNK/NF–κB pathways.

Acute respiratory distress syndrome (ARDS) is an inflammatory response to both pulmonary and extra–pulmonary stimuli, characterized by acute onset of new or worsening respiratory dysfunction. Despite improvements in intensive care with optimal ventilation support and fluid balance, the mortality of patients with ARDS remains above 30%^1^,^2^. Diffuse pulmonary endothelial cell injury that results in impairment of the alveolar–capillary barrier, and increase in microvascular endothelial permeability, are considered central to the pathogenesis of ARDS^3^.

The renin–angiotensin system (RAS) is a complex hormonal system and a pivotal regulator in maintaining homeostasis of blood pressure and electrolyte balance; RAS also has an important role in inflammation^4^. Abnormal activation of the RAS is involved in the pathogenesis of cardiovascular, renal, and lung diseases^5^,^6^,^7^. Angiotensin–converting enzyme (ACE) 2, a homologue of ACE, is a recently discovered component of the RAS^8^. In contrast to ACE which converts angiotensin (Ang) I (AngI) to generate AngII, ACE2 reduces the generation of AngII by catalyzing the conversion of AngII to Ang–(1–7), which attenuates the vasoconstrictive, proliferative, and inflammatory effects of AngII. Hence, ACE2 has a pertinent role in the anti–inflammatory RAS–ACE2–Ang–(1–7) axis, as it counteracts the pro–inflammatory effects of the ACE–AngII axis^9^,^10^.

The article "Angiotensin-converting enzyme 2/angiotensin-(1–7)/Mas axis prevents lipopolysaccharide–induced apoptosis of pulmonary microvascular endothelial cells by inhibiting JNK/NF–κB pathways" was retracted in 2026. Reasons: plagiarized images; duplicated images; overlap with other authors' work; overlap with earlier publications.

ACE2 is a membrane–associated aminopeptidase in vascular endothelia, renal and cardiovascular tissues, and epithelia of the small intestine and testes^11^,^12^. ACE2 is also broadly expressed in almost all kinds of cell types in the lung, including endothelial and smooth muscle cells of blood vessels, types I and II alveolar epithelial cells, and bronchial epithelial cells. There is also evidence that ACE2 has an important role in the development of ARDS. In fact, ACE2 levels positively correlated with severe acute respiratory syndrome (SARS) coronavirus infection of human airway epithelia^13^. In addition, ACE2–deficient mice suffered more aggravated lung injury compared with wild–type mice in models of ARDS, whereas therapy with recombinant ACE2 improved ARDS in *Ace2*–knockout, especially in wild–type mice^14^. All these findings suggest that ACE2 may prevent lung injury and may be useful as a therapeutic agent targeting ARDS.

Several studies have shown that mitogen–activated protein kinases (MAPKs) may have key roles in acute lung injury. For example, inhibition of p38 MAPK phosphorylation and activity protects against pulmonary infiltration of leukocytes as well as lung edema^15^. Activation of p38 MAPK appears to be an important upstream signaling event associated with tumor necrosis factor (TNF)–α–induced barrier failure in the pulmonary endothelial monolayer^16^. Furthermore, inhibition of p38 MAPK, but not extracellular signal regulated kinase (ERK), significantly attenuated TNF–α–induced increase of endothelial permeability^17^. The MAPK pathway also mediates regulation of *Ace2* mRNA expression in rat aortic vascular smooth muscle cells^18^.

Lipopolysaccharide (LPS), released from the gram–negative bacterial cell wall, contributes to pulmonary inflammation and sepsis that leads to ARDS^19^,^20^. Upon recognition by toll–like receptor 4 (TLR4) on the cellular surface, LPS activates nuclear factor–κB (NF–κB) and MAPKs cascades, leading to the release of pro–inflammatory cytokines such as interleukin (IL)–1, IL–6, and TNF–α^21^,^22^,^23^. TLR4–NF–κB signaling regulates the severity of acute lung injury (ALI)^24^. p38 MAPK, ERK, and NF–κB are activated during LPS–induced lung injury^25^. Inhibition of ERK prevents LPS–induced inflammation by suppressing NF–κB transcription activity^26^,^27^. Inhibition of p38 MAPK attenuates pulmonary inflammatory responses induced by LPS and reduces the activation of NF–κB^28^.

The article "Angiotensin-converting enzyme 2/angiotensin-(1–7)/Mas axis prevents lipopolysaccharide–induced apoptosis of pulmonary microvascular endothelial cells by inhibiting JNK/NF–κB pathways" was retracted in 2026. Reasons: plagiarized images; duplicated images; overlap with other authors' work; overlap with earlier publications.

ACE2 was found to be beneficial for both cardiac and pulmonary protection. For instance, ACE2 inhibited cardiac fibrosis through a reduction in ERK phosphorylation^29^. Telmisartan protects against heart failure by upregulating the ACE2/ANG–(1–7)/Mas receptor axis, by inhibiting expression of phospho–p38 MAPK, phospho–c–jun N–terminal kinases (JNK), phospho–ERK, and phospho–MAPK–activated protein kinase–2^30^. Furthermore, upregulating ACE2 can lessen lung injury^31^, and ACE2 or angiotensin–(1–7) has an important role in preventing ARDS^32^. However, whether upregulation of the ACE2/Ang–(1–7)/Mas axis prevents LPS–induced apoptosis of pulmonary microvascular endothelial cells by inhibiting the MAPKs/NF–κB pathways remains unknown.

For the present study, we investigated whether upregulation of ACE2 expression may prevent LPS–induced pulmonary inflammation and cytotoxicity by way of the MAPK/NF–κB signal pathway.

## Methods

### Reagents

LPS from *Escherichia coli*, (O127:B8) was purchased from Sigma–Aldrich (St. Louis, MO, USA). Rabbit anti–ACE, anti–ACE2, and anti–p65, and mouse anti–phospho–p65 and anti–IκBα antibodies were procured from Santa Cruz Biotechnology (Delaware, CA, USA). Rabbit anti–p38 MAPK, anti–phospho–p38 MAPK, anti–ERK1/2, anti–phospho–ERK1/2, anti–stress–activated protein kinase (SAPK)/JNK, anti–phospho–SAPK/JNK, horseradish peroxidase (HRP)–conjugated secondary antibody goat anti–rabbit IgG, and horse anti–mouse IgG antibodies were all purchased from Cell Signaling Technology (Danvers, MA, USA). TNF–α and IL–1β kits were purchased from Invitrogen (Eugene, OR, USA). AngII and Ang–(1–7) enzyme–linked immunosorbent assay (ELISA) kits came from Kamiya Biomedical (Seattle, WA, USA). Mas receptor blocker A779 was obtained from AbBiotech (San Diego, CA, USA). SB203580 (a specific inhibitor of p38 MAPK), PD98059 (a specific inhibitor of ERK1/2) and SP600125 (a specific inhibitor of JNK) were all purchased from Santa Cruz Biotechnology (Delaware, CA, USA).

### Animals

Sprague–Dawley rats weighing 200–250 g were obtained from the Department of Laboratory Animal Science of Fudan University, Shanghai, China. All animals were handled in accordance with the protocol approved by the Ethics Committee of Animal Research at the College of Medicine, Shanghai Jiaotong University, Shanghai, China.

### Cell culture

Isolation and culture of pulmonary microvascular endothelial cells (PMVECs) were performed as described previously^3^. Briefly, the rats were euthanized after intraperitoneal injection of pentobarbital sodium. Thoracotomy was performed and the lung circulatory system was perfused by injection of 50 mL ice–cold phosphate buffered saline (PBS) via the right ventricle. The lungs were removed and washed with 30 mL ice–cold serum–free Dulbecco's modified Eagle's medium (DMEM, Sigma–Aldrich, St. Louis, MO, USA).

The article "Angiotensin-converting enzyme 2/angiotensin-(1–7)/Mas axis prevents lipopolysaccharide–induced apoptosis of pulmonary microvascular endothelial cells by inhibiting JNK/NF–κB pathways" was retracted in 2026. Reasons: plagiarized images; duplicated images; overlap with other authors' work; overlap with earlier publications.

The pleura were carefully cut away and discarded, and then sections (1 mm) were cut from the outer edge of the remaining lung tissue and trimmed into small pieces. These lung tissue pieces were then inserted into the glass pellets (Costar, Cambridge, MA) and rinsed in endothelial cell medium (ScienCell Research, Carlsbad, CA, USA) supplemented with 20% fetal calf serum, 100 U/mL penicillin/streptomycin, and 2.5 g/mL amphotericin B. The glass pellets were incubated in humidified air with 5% CO_2_ for 60 h, and the culture media were replaced every 3 days.

The cells at 80–90% confluence were harvested by treating with 0.25% trypsin– ethylenediaminetetraacetic acid (EDTA; Gibco, Grand Island, NY, USA) and subcultured at 1:2 ratios. Cobblestone morphology and immunostaining with rabbit anti–human factor VIII, anti–rat CD31 (Boster, Wuhan, China), and fluorescein isothiocyanate (FITC)–*Bandeiraea simplicifolia* isolectin (BSI; Santa Cruz, Delaware, CA, USA) were used to identify the endothelial cells. The third to fifth cell passages were used for the following experiments.

### Generation of recombinant *Ace2* and small hairpin RNA (shRNA)–*Ace2* lentiviruses

Total RNA was extracted from rat PMVECs and reversely transcribed into cDNA using M–MLV reverse transcriptase (Takara BIO, Japan). The cDNA was used to amplify the *Ace2* coding sequence with the following primers: forward, 5′–GCTCTAGAGCCACCATGTCAAGCTCCTGCTGGC–3′ and reverse, 5′– CGGGATCCTTAGAATGAAGTTTGAGC. Three shRNA sequences targeting the rat *Ace2* coding region (homologous to nt 1089–1107, 1152–1170, and 1582–1600 of *Ace2* mRNA, respectively) were designed: small interfering RNA (siRNA)1–*Ace2* (5′–GGTCACAATGGACAACTTC–3′); siRNA2–*Ace2* (5′–GCATATGCCAAGCAACCTT–3′); and siRNA3–ACE2 (5′–GCTCTTTGTCAAGCAGCTA–3′). An invalid RNA interference (RNAi) sequence (5′–GAAGCCAGATCCAGCTTCC–3′) was used as the negative control. The corresponding oligonucleotide templates of the shRNAs were chemically synthesized. The *Ace2* PCR products were purified and ligated to a lentiviral pcDNA–CMV–copGFP cDNA vector and the synthesized shRNA–*Ace2* to pSIH1–H1–copGFP shRNA (System Biosciences, CA, USA). Each ligation mixture was transformed into competent *E. coli* strain DH5α, and the resultant plasmids were confirmed by sequencing.

The article "Angiotensin-converting enzyme 2/angiotensin-(1–7)/Mas axis prevents lipopolysaccharide–induced apoptosis of pulmonary microvascular endothelial cells by inhibiting JNK/NF–κB pathways" was retracted in 2026. Reasons: plagiarized images; duplicated images; overlap with other authors' work; overlap with earlier publications.

In accordance with the manufacturer's instructions, the vectors carrying *Ace2* or *Ace2* shRNA and lentivirus package plasmids were co–transfected into 293 T producer cells using Lipofectamine 2000 (Invitrogen, Carlsbad, CA, USA). The supernatants were collected 48 h later. Total RNA and protein were extracted to determine ACE2 mRNA and protein and to select a recombinant shRNA lentivirus with the most sufficient siRNA. Viral titer was evaluated by gradient dilution. The recombinant lentiviruses were named LV–*Ace2* and LV–shRNA–*Ace2*.

### Lentiviral transduction

One day after seeding, PMVECs cells were infected with LV–*Ace2* or LV–shRNA–*Ace2* and diluted at a multiplicity of infection (MOI) of 20 in endothelial cell medium, which was refreshed 24 h later. The infection efficiency was assessed by fluorescence microscopy 96 h after infection.

One hundred microliters of PMVECs, normal or lentivirus–infected (LV–*Ace2* or LV–shRNA–*Ace2*), were seeded into 96–well plates (1 × 10^4^ cells/well) and incubated with serum–free DMEM for 24 h. PMVECs, whether normal or infected, were then pretreated (or not) with 100 nM A779 for 2 h and then stimulated (or not) with 1 mg/mL LPS for 48 h as follows: (1) normal cells in PBS and untreated (control); (2) normal cells, treated with A779, without LPS (A779); (3) normal cells, treated with LPS only (LPS); (4) normal cells, treated with A779 and also LPS (A779 + LPS); (5) cells infected with the empty control virus, receiving LPS only (Lv–control + LPS); (6) cells infected with RNAi (negative control or NC) receiving LPS only (Lv–NC + LPS); (7) cells infected with shRNA–*Ace2*, receiving LPS only (shACE2 + LPS); (8) cells infected with LV–*Ace2*, receiving LPS only (ACE2 + LPS); and (9) cells infected with LV–*Ace2*, receiving A779 prior to LPS (ACE2 + A779 + LPS).

For further experiments using the specific MAPK inhibitors, normal cells and cells infected with shRNA–*Ace2* or LV–*Ace2* were pre–incubated with either 10 μM SB203580, 20 μM PD98059, or 20 μM SP600125, for 2 hours before exposure to LPS.

### Apoptosis assay

Apoptosis was determined using an annexin V–FITC apoptosis detection kit (BD, Franklin Lakes, NJ, USA) in accordance with the manufacturer's protocol. In brief, the cells were harvested, washed 3 times with PBS, centrifuged at 2000 × *g* for 5 min, and resuspended in 500 μL of binding buffer (0.1 M Hepes/NaOH, 1.4 M NaCl, 25 mM CaCl_2_, pH 7.4) to a final concentration of 1 × 10^6^ cells/mL. After incubation with 5 μL of annexin V–FITC for 10 min and 5 μL of propidium iodide for 5 min at room temperature, the cell suspension was subjected to flow cytometry on a FACSCalibur (BD, Franklin Lakes, NJ, USA) and detected at excitation wavelength 488 nm. Data were analyzed using CellQuest Pro software (BD, Franklin Lakes, NJ, USA).

The article "Angiotensin-converting enzyme 2/angiotensin-(1–7)/Mas axis prevents lipopolysaccharide–induced apoptosis of pulmonary microvascular endothelial cells by inhibiting JNK/NF–κB pathways" was retracted in 2026. Reasons: plagiarized images; duplicated images; overlap with other authors' work; overlap with earlier publications.

### Detection of cytokine secretions

The culture supernatants of each group were collected and frozen at −20°C, and IL–1β, TNF–α, AngII and Ang–(1–7) concentrations in the supernatants were assayed by sandwich ELISA. Briefly, 96–well plates were coated with the monoclonal antibody specific to IL–1β, TNF–α, AngII, or Ang–(1–7) supplied in the ELISA kit. ELISAs were performed in accordance with the manufacturer's instructions. Finally, the absorbance at 450 nm was measured using a micro–plate reader (Bio–Rad Laboratories, Hercules, CA, USA). The concentrations were extrapolated from the standard curve obtained from the same plate.

### Western blot analysis

Total protein was extracted from the cells using M–PER Mammalian Protein Extraction Reagent (Pierce, IL, USA). The protein concentration was determined with a bicinchoninic acid protein assay kit (Pierce, USA), and equal amounts of protein (25 μg) were run on a 12% SDS–PAGE gel and transferred onto nitrocellulose membranes. The membranes were blocked with 5% skim milk in Tris–buffered saline (10 mM Tris, 150 mM NaCl, pH7.4)/0.1% Tween 20 (TBST) at room temperature for 2 h. The blots were probed with a primary antibody against rat ACE (1:400), ACE2 (1:500), ERK1/2 (1:400), SAPK/JNK (1:500), p38 MAPK (1:600), IκBα (1:500), phosphorylated P65 (1:300), P65 (1:500) and β actin (1:1000). After 3 washes with TBST, the blots were incubated in secondary HRP–conjugated anti–mouse/rabbit IgG. After washing with TBST 3 times, the membranes were developed with a chemiluminescence (ECL) detection kit and imaged with X–ray films. Beta actin was used as an endogenous reference for normalization.

### Statistical analyses

All data are presented as mean ± standard deviation (SD). Statistical analyses were performed with the Prism software package (GraphPad v5, San Diego, CA, USA). Data were analyzed using one–way ANOVA and then the Newman–Keuls test for multiple comparisons. A *P*–value less than 0.05 was accepted as statistically significant.

## Results

### Effects of ACE2 and Mas–receptor antagonist A779on LPS–induced apoptosis in PMVECs

The rate of apoptosis of PMVECs in the LPS group (exposed to LPS for 48 h; 55.07%), was significantly higher than that of the PBS control group (6.43%; *P* < 0.05; Fig. 1A). For cells infected with LV–*Ace2* receiving LPS (ACE2 + LPS group) the rate of apoptosis was 37.60% (*P* < 0.05), but this was significantly lower than that of PMVECs infected with shRNA–ACE2 treated with LPS (shACE2 + LPS group; 85.85%; *P* < 0.05).

The article "Angiotensin-converting enzyme 2/angiotensin-(1–7)/Mas axis prevents lipopolysaccharide–induced apoptosis of pulmonary microvascular endothelial cells by inhibiting JNK/NF–κB pathways" was retracted in 2026. Reasons: plagiarized images; duplicated images; overlap with other authors' work; overlap with earlier publications.

In normal PMVECs stimulated with LPS, the apoptosis rate of those given the A779 pretreatment (A779 + LPS group; 89.55%) was significantly higher than that of the cells treated with LPS only (LPS; 55.07%; *P* < 0.05; Fig. 1B). However, the apoptosis rate of cells infected with LV–*Ace2* that received pretreatment of A779 prior to LPS (ACE2 + A779 + LPS group; 53.80%) was significantly lower than that of the A779 + LPS group (*P* < 0.05), although there was no significant difference between the ACE2 + A779 + LPS group (53.80%) and the LPS group (55.07%).

### Effects of ACE2 and Mas–receptor antagonist A779 on cytokine secretion in PMVECs

The IL–1β and TNF–α levels in the supernatants of cultured PMVECs that were exposed to LPS for 48 h were significantly higher as compared with control group. (Fig. 2A, 2C). LPS–induced IL–1β and TNF–α secretions were significantly inhibited by ACE2 overexpression, but further promoted by ACE2 knockdown.

In PMVECs exposed to LPS, pretreatment with A779 caused a significant increase in IL–1β and TNF–α secretions, which were markedly attenuated by ACE2 overexpression (Fig. 2B, 2D). However, there was no significant difference between ACE2 + A779 + LPS and LPS–treated cells in the levels of cytokines in the supernatants. These results indicate that ACE2 suppressed the LPS–induced inflammatory response in PMVECs, and the Mas–receptor antagonist effectively prevented this protective effect.

### Effects of ACE2 and Mas–receptor antagonist A779 on AngII/Ang–(1–7) secretion in PMVECs

The AngII levels in supernatants of the LPS group (20.04 ± 1.92 ng/mL) were significantly higher than that of the PBS control group (10.99 ± 4.03 ng/mL; *P* < 0.05), but the Ang–(1–7) levels in the LPS group were only slightly higher (15.49 ± 3.41 ng/mL) than that of the PBS group (12.30 ± 2.40 ng/mL; *P* > 0.05).

For cells infected with LV–*Ace2* receiving LPS (ACE2 + LPS group), AngII secretion (12.79 ± 2.42 ng/mL) was significantly less than that of the normal cells receiving LPS (LPS group; 20.04 ± 1.92 ng/mL), but AngII levels were significantly higher in PMVECs infected with shRNA–*Ace2* treated with LPS (shACE2 + LPS group; 27.29 ± 3.97 ng/mL) compared with the LPS group (*P* < 0.05).

In contrast, Ang–(1–7) levels in PMVECs infected with LV–*Ace2* receiving LPS (ACE2 + LPS group; 31.20 ± 4.75 ng/mL; *P* < 0.05) were significantly higher than that of the LPS group (15.49 ± 3.41 ng/mL), and also that of the shRNA–ACE2 + LPS group (14.81 ± 2.55 ng/mL; *P* < 0.05; Fig 3A, 3C).

In normal PMVECs exposed to LPS, the AngII levels of those pretreated with A779 (A779 + LPS group; 31.87 ± 4.69 ng/mL) were significantly higher than that of the cells treated with LPS only (20.04 ± 1.92 ng/mL; *P* < 0.05). The AngII levels of cells infected with LV–*Ace2* that received pretreatment of A779 prior to LPS (ACE2 + A779 + LPS group; 15.50 ± 0.60 ng/mL) were significantly lower than that of the A779 + LPS group (31.87 ± 4.69 ng/mL; *P* < 0.05).

The article "Angiotensin-converting enzyme 2/angiotensin-(1–7)/Mas axis prevents lipopolysaccharide–induced apoptosis of pulmonary microvascular endothelial cells by inhibiting JNK/NF–κB pathways" was retracted in 2026. Reasons: plagiarized images; duplicated images; overlap with other authors' work; overlap with earlier publications.

However, the levels of Ang–(1–7) in normal PMVECs treated with A779 and LPS (A779 + LPS group; 10.12 ± 2.80 ng/mL) were slightly less than these levels in the LPS group (15.49 ± 3.41; *P* > 0.05), and those of the ACE2 + A779 + LPS group (16.23 ± 5.17 ng/mL) were only slightly higher (*P* > 0.05; Fig 3B, 3D).

### Effects of ACE2 and Mas–receptor antagonist A779 on the ACE2/ACE ratio in PMVECs

Relative to the normal PMVECs in PBS (control group), in those stimulated with LPS for 48 h (LPS group) the ACE levels were higher and the ACE2 levels were lower, and therefore the ACE2/ACE ratio was significantly lower (Fig. 4A). However, in cells infected with LV–*Ace2* receiving LPS only (ACE2 + LPS group), the ACE2/ACE ratio was comparable to the control group (*P* > 0.05). In contrast, cells infected with shRNA–*Ace2* receiving LPS only (shACE2 + LPS group), the ratio of ACE2/ACE ratio was lower than that of the LPS group.

Compared with the ACE2/actin and ACE/actin levels of the LPS group (0.2924 and 0.6918, respectively), both of these were significantly lower in normal PMVECs treated with A779 prior to LPS (A779 + LPS group; 0.2187 and 0.5462; *P* < 0.05 for both). The ACE2/ACE ratio was also notably lower in the A779 + LPS group compared to the control group, but was not significantly different from that of the LPS group (Fig. 4B). In addition, compared with the ACE2/actin and ACE/actin levels of the normal cells treated with A779 and LPS (A779 + LPS group; 0.2187 and 0.5462, respectively), in the cells infected with LV–*Ace2* and treated with both A779 and LPS (ACE2 + A779 + LPS group), ACE2/actin was significantly higher (0.3733; *P* < 0.05) while ACE/actin (0.4707) was similar (*P* > 0.05). As a result, the ratio of ACE2/ACE was much higher in the A779 + ACE2 + LPS group.

### Effects of ACE2 and Mas–receptor antagonist A779 on the MAPKs phosphorylation in PMVECs

The western blot results showed that after normal PMVECs were incubated with LPS for 48 h (LPS group), phosphorylation levels of ERK1/2, p38, and SAPK/JNK were significantly higher compared with the untreated control group (Fig 5A, 5C, 5E). Compared with the LPS group, PMVECs transduced with *Ace2* and incubated with LPS (ACE2 + LPS group) had lower levels of phosphorylated p38 and SAPK/JNK, but levels of ERK1/2 phosphorylation were not markedly less. In contrast, compared with the LPS group, PMVECs transduced with shRNA–*Ace2* and incubated with LPS (shACE2 + LPS group) had significantly higher ERK1/2 phosphorylation levels, but levels of phosphorylated p38 and SAPK/JNK were similar.

The article "Angiotensin-converting enzyme 2/angiotensin-(1–7)/Mas axis prevents lipopolysaccharide–induced apoptosis of pulmonary microvascular endothelial cells by inhibiting JNK/NF–κB pathways" was retracted in 2026. Reasons: plagiarized images; duplicated images; overlap with other authors' work; overlap with earlier publications.

Pretreatment with A779 in LPS–exposed cells (A779 + LPS group) was associated with significantly higher phosphorylation levels of all three MAPK pathways relative to cells of the LPS group. Whereas compared with the A779 + LPS group, the levels of phosphorylated p38 and SAPK/JNK phosphorylation in the ACE2 + A779 + LPS group were markedly lower (*P* < 0.05), there was no obvious difference in these levels between the ACE2 + A779 + LPS and LPS groups (*P* > 0.05; Fig. 5B, D, F). Furthermore, compared with the A779 + LPS group, the ERK1/2 phosphorylation level was only slightly less in the ACE2 + A779 + LPS group (*P* > 0.05), but significantly higher than that of the LPS group and the phosphorylation level in the A779 + LPS group was still more enhanced than in LPS group (*P* < 0.05).

In addition, the levels of phosphorylated ERK1/2 in the A779 + LPS group were approximately the same as that of the shACE2 + LPS group (*P* > 0.05), while the levels of phosphorylated p38 and SAPK/JNK were significantly higher (*P* < 0.05).

### Effects of ACE2 and Mas–receptor antagonist A779 on NF–κB p65 phosphorylation and IκBα expression in PMVECs

The phosphorylation of NF–κB p65 and expression of IκBα were examined by western blot (Fig. 6). LPS stimulation resulted in significantly increased level of NF–κB p65 phosphorylation and decreased level of IκBα expression in normal PMVECs. In the cells infected with LV–*Ace2* and stimulated with LPS (ACE2 + LPS group), the NF–κB p65 phosphorylation level was significantly lower and IκBα expression level significantly higher than that in PMVECs stimulated with LPS only. In contrast, compared with the LPS group, PMVECs transduced with shRNA–*Ace2* and stimulated with LPS (shACE2 + LPS group) had significantly higher NF–κB p65 phosphorylation levels and lower IκBα expression levels.

The phosphorylation levels of NF–κB p65 were significantly higher and the IκBα levels lower in the cells stimulated with LPS and pretreated with A779 (A779 + LPS group) compared with the LPS group. The phosphorylated NF–κB p65 levels in the ACE2 + A779 + LPS group were significantly higher than that of the LPS group, but were not significantly different from the ACE2 + A779 + LPS and A779 + LPS groups. The IκBα levels in the ACE2 + A779 + LPS group was approximately similar to that of the LPS group, but was significantly increased compared with the A779 + LPS group.

The article "Angiotensin-converting enzyme 2/angiotensin-(1–7)/Mas axis prevents lipopolysaccharide–induced apoptosis of pulmonary microvascular endothelial cells by inhibiting JNK/NF–κB pathways" was retracted in 2026. Reasons: plagiarized images; duplicated images; overlap with other authors' work; overlap with earlier publications.

### Effects of MAPKs specific inhibitors on LPS–induced apoptosis in PMVECs

To clarify whether inhibition of MAPK activation influences the effects of ACE2 and the Mas–receptor antagonist on LPS–induced PMVEC apoptosis, the cells were pre–incubated with MAPK signaling pathway specific inhibitors SB203580, PD98059, or SP600125 before LPS stimulation (Fig. 7). Compared with the apoptosis level of 55.07% in the LPS group, only pretreatment with SP600125, with or without A779 pretreatment, significantly inhibited LPS–induced apoptosis in normal, ACE2, or shACE2 transduced PMVECs, with apoptosis levels of 15.33%, 22.97%, 22.60% and 23.20% in the ACE2 + LPS + SP600125, shACE2 + LPS + SP600125, A779 + LPS + SP600125 and ACE2 + A779 + LPS + SP600125 groups, respectively (*P* < 0.05).

The apoptosis of cells infected with LV–*Ace2* and stimulated with LPS was not significantly increased by SB203580 or PD98059 pretreatment (37.60% in the ACE2 + LPS group compared to 49.64% and 48.08% in the ACE2 + LPS + SB203580 and ACE2 + LPS + PD98059 groups, respectively, *P* > 0.05). The apoptosis levels of cells infected with LV–*Ace2* and pretreated with both A779 and SB203580, or PD98059 prior to LPS stimulation were significantly higher than that of the ACE2 + A779 + LPS group, with 87.46% and 85.68% in the ACE2 + A779 + LPS + SB203580 and ACE2 + A779 + LPS + PD98059 groups, respectively, compared with 53.80% in the ACE2 + A779 + LPS group (*P* < 0.05).

SB203580 or PD98059 pre–treatment did not affect the apoptosis of cells infected with shACE2 or the normal cells pretreated with A779 before LPS stimulation, with 79.35% in the shACE2 + LPS + SB203580, 77.40% in the shACE2 + LPS + PD98059, 85.85% in the shACE2 + LPS, 89.87% in the A779 + LPS + SB203580 and 84.03% in the A779 + LPS + PD98059 groups, compared with 89.55% in the A779 + LPS group (*P* > 0.05).

### Effects of MAPKs signaling specific inhibitors on LPS–induced cytokine secretion in PMVECs

In cells infected with LV–*Ace2* and stimulated with LPS (ACE2 + LPS group), pretreatment with specific MAPK signaling inhibitors did not affect LPS–induced IL–1β or TNF–α secretions (Fig. 8A, 8B). In contrast, pre–treatment with MAPK signaling inhibitors, especially the pretreatment with SP600125 in the PMVECs transduced with shRNA–*Ace2* and stimulated with LPS (shACE2 + LPS group), significantly suppressed cytokine secretion (Fig. 8C, 8D).

In PMVECs exposed to LPS, pretreatment with A779 significantly increased, but SB203580 and PD98059 slightly reduced and SP600125 significantly attenuated, IL–1β and TNF–α secretions (Fig. 8E, 8F). In addition, pre–incubation with SB203580 or PD98059 did not affect LPS–induced IL–1β or TNF–α secretions in the cells infected with LV–*Ace2* and pretreated with A779 prior to LPS stimulation (ACE2 + A779 + LPS group). LPS–induced IL–1β and TNF–α secretions in the ACE2 + A779 + LPS group were significantly inhibited by pre–incubation with SP600125 (Fig. 8G, 8H).

The article "Angiotensin-converting enzyme 2/angiotensin-(1–7)/Mas axis prevents lipopolysaccharide–induced apoptosis of pulmonary microvascular endothelial cells by inhibiting JNK/NF–κB pathways" was retracted in 2026. Reasons: plagiarized images; duplicated images; overlap with other authors' work; overlap with earlier publications.

## Discussion

In the present study, we investigated the effect of overexpressed or shRNA–inhibited *Ace2* on LPS–induced injury in lentivirus–transduced PMVECs. We found that ACE2 overexpression attenuated apoptosis and IL–1β and TNF–α secretion caused by LPS stimulation. Both *Ace2* deletion and Mas receptor inhibition exhibited almost similar deteriorating effects on LPS–induced damage and cytokine secretion, by blocking ACE2 overexpression. Therefore, the protective effects of ACE2 overexpression on LPS–induced apoptosis and the inflammatory response may be through regulation of the ACE2/ACE/AngII/Ang–(1–7)/Mas receptor.

In fact, ACE2 acts as a counter–regulator of ACE in regulating the production of AngII and Ang–(1–7)^33^. In addition, SARS–CoV infections caused a downregulation of ACE2 expression in lungs, while ACE2 treatment protected mouse lungs from severe acute injury^13^. It is also noted that ACE2 expression in lung tissue was downregulated in a mouse ARDS model induced by acid aspiration, endotoxin, and peritoneal sepsis^14^. In the same study, loss of ACE2 expression in mutant mice resulted in more severe lung injury, enhanced vascular permeability, increased lung edema, and worsened lung function.

We found that AngII levels in cell supernatants were higher after LPS stimulation than before LPS stimulation. In addition, ACE2 overexpression reversed the imbalance of ACE2/ACE, and significantly reduced AngII and increased Ang(1–7) levels, thus reducing LPS–induced apoptosis and inflammation. In contrast, the shRNA–inhibited ACE2 expression aggravated the imbalance of ACE2/ACE, markedly increased AngII and decreased Ang(1–7) levels, to promote apoptosis and the inflammatory response caused by LPS exposure.

The Mas receptor blocker effectively abolished the protective effects of *Ace2* transgenesis but the imbalance of ACE2/ACE was not affected. Treatment with Mas receptor blocker A779 before LPS stimulation also significantly increased AngII but had no obvious influence on Ang(1–7) levels. This may be ascribed to the significant suppression of ACE2 expression by the Mas receptor blocker. Therefore, the protective effect of ACE2 on LPS–induced PMVEC injury may be via regulation of the ACE2/ACE/AngII/Ang–(1–7)/Mas receptor. In fact, many reports suggest that AngII exerts pro–inflammatory effects by inducing the release of cytokines, chemokines, adhesion molecules, growth factors, and reactive oxygen species through AT1 receptors^34^,^35^. AngII can also significantly induce apoptosis of pulmonary endothelial cells through the AT1 receptor, leading to damage in epithelial barrier function and increased permeability^36^.

The article "Angiotensin-converting enzyme 2/angiotensin-(1–7)/Mas axis prevents lipopolysaccharide–induced apoptosis of pulmonary microvascular endothelial cells by inhibiting JNK/NF–κB pathways" was retracted in 2026. Reasons: plagiarized images; duplicated images; overlap with other authors' work; overlap with earlier publications.

On the other hand, Ang–(1–7) binds to the specific G–protein–coupled receptor Mas to counteract AngII function (i.e., vasodilatory, anti–growth, and anti–proliferative effects). Overexpression of Ang(1–7) prevents bleomycin–induced lung injury, and blockade of the Mas receptor abolishes the beneficial effects of Ang(1–7) against monocrotaline–induced pulmonary hypertension^37^. Ang(1–7) attenuates ventilator– or acid aspiration–induced lung injury and barrier failure of PMVECs, but this effect is again blocked by Mas receptor blockers^38^.

Moreover, experimental results also indicate that unbalanced AngII/Ang(1–7) is associated with the development of ARDS, and a change in AngII/Ang(1–7) is closely related to the ratio of ACE2/ACE. In bronchoalveolar lavage fluid (BALF) of ventilated animals exposed to LPS, ACE2 activity is reduced, whereas ACE activity is enhanced, and these changes are in accord with enhanced BALF levels of AngII and reduced levels of Ang(1–7)^32^. After hind–limb ischemia–reperfusion, an imbalance in ACE2/ACE in local lung tissue is accompanied by changes in AngII/Ang(1–7)^31^. Thus, we believe that an imbalance in ACE2/ACE/AngII/Ang–(1–7)/Mas receptor mediates lung injury, and regulation of RAS homeostasis by ACE2 may improve LPS–induced lung injury.

The activation of MAPKs pathways has a key role in progression to acute lung injury but has not been fully elucidated in PMVECs after exposure to LPS^15^,^16^. In the present study, we found that ACE2 overexpression significantly blocked LPS–induced activation of the p38 and JNK pathways, which was strikingly prevented by administration of the Mas receptor blocker. This suggests that ACE2 is protective against LPS–induced apoptosis of PMVECs and inflammation, perhaps through the Ang–(1–7)/Mas pathway to modulate p38 and JNK phosphorylation. On the other hand, shRNA–ACE2 enhanced LPS–induced ERK phosphorylation but had no influence on p38 and JNK phosphorylation, whereas LPS–mediated increased ERK phosphorylation was not affected by ACE2 overexpression in cells pretreated with the Mas receptor blocker. These results suggest that inhibited ACE2 aggravated LPS–induced PMVEC apoptosis and inflammation mainly through the AngII/AT1 pathway to enhance ERK phosphorylation. In fact, activation of p38 MAPK and ERK is associated with TNF–α–induced increase of permeability in pulmonary endothelial cells, and the proliferation and survival of lung endothelial cells to maintain endothelial monolayer integrity may be by way of activating p38 MAPK^39^. Bleomycin induces cell apoptosis through the JNK phosphorylation pathway in alveolar epithelial cells (AECs)^40^. In addition, ACE2 regulates the balance of AngII/Ang(1–7) to inhibit apoptosis of alveolar epithelial cells through blockade of JNK phosphorylation^41^.

The article "Angiotensin-converting enzyme 2/angiotensin-(1–7)/Mas axis prevents lipopolysaccharide–induced apoptosis of pulmonary microvascular endothelial cells by inhibiting JNK/NF–κB pathways" was retracted in 2026. Reasons: plagiarized images; duplicated images; overlap with other authors' work; overlap with earlier publications.

We also performed additional experiments to determine whether the ACE2/Ang–(1–7)/Mas axis prevents the LPS–induced inflammatory response and apoptosis of rat PMVECs via inhibition of p38 and JNK phosphorylation. We found that the protective effect of ACE2 overexpression on LPS–induced apoptosis was enhanced by the JNK inhibitor and deteriorated by p38 and ERK inhibition. The JNK inhibitor markedly reduced apoptosis and cytokine secretion in PMVECs with *Ace2* deletion and pretreatment with the Mas receptor antagonist. The Mas receptor antagonist abolished the protective effect of ACE2, which was aggravated by p38 and ERK inhibitors but was reversed by JNK inhibition. Therefore, these data suggest that ACE2/Ang–(1–7)/Mas may have a protective effect on LPS–induced apoptosis and inflammation in PMVECs, mainly through inhibition of the JNK pathway.

In the present study, we found that ACE2 overexpression significantly inhibited LPS–induced activation of the NF–κB and degradation of IκBα protein, which was strikingly reversed by the Mas receptor antagonist. In addition, both the ACE2 downregulation and A779 pretreatment enhanced NF–κB phosphorylation and further degraded IκBα protein, suggesting that the NF–κB pathway is also important in the prevention of ACE2/Ang–(1–7)/Mas from LPS–induced PMVEC apoptosis and inflammation. In fact, NF–κB binds to IκBα in the cytoplasm, but once dissociated from IκBα, NF–κB is activated and translocates into the nucleus to upregulate transcription of several inflammatory genes^45^,^46^. The NF–κB cascade is pivotal to the intracellular signaling pathway involved in apoptosis and the inflammatory response, and activation of NF–κB is central to the regulation of pulmonary inflammation and involved in the pathogenesis of ARDS^42^,^43^,^44^. LPS–induced lung injury is associated with activation of MAPKs and NF–κB signaling pathways^47^; the inhibition of ERK or p38 protects against LPS–induced lung injury by inhibiting the NF–kB pathway^28^,^48^. Pretreatment with Ang–(1–7) prevents AngII–induced lung fibroblast apoptotic resistance by inhibiting the MAPK/NF–kB pathway^49^.

In conclusion, our results suggest that abnormal activation of RAS with unbalanced AngII/Ang(1–7) levels, induced by the imbalance of ACE2/ACE expression, is closely related to LPS–mediated apoptosis and inflammation in PMVECs. Furthermore, ACE2 exerts protective effects on LPS–induced apoptosis and inflammation in PMVECs through suppression of the JNK/NF–kB signaling pathways. Our findings imply that ACE2 may be applied to improve LPS–induced lung injury via regulation of the ACE2/ACE/AngII/Ang–(1–7)/Mas receptor, by inhibiting the JNK/NF–kB signaling pathway, and that upregulation of the ACE2/Ang–(1–7)/Mas axis and inhibition of JNK/NF–kB activation may be an effective therapeutic strategy against ARDS in clinic.

The article "Angiotensin-converting enzyme 2/angiotensin-(1–7)/Mas axis prevents lipopolysaccharide–induced apoptosis of pulmonary microvascular endothelial cells by inhibiting JNK/NF–κB pathways" was retracted in 2026. Reasons: plagiarized images; duplicated images; overlap with other authors' work; overlap with earlier publications.

A limitation of this study is that the results did not address the crosstalk between MAPK and NF–kB signaling pathways. Further studies are necessary to investigate possible crosstalk among the intracellular signaling pathways involved in the effects of Ang(1–7)/Mas receptor on LPS–induced PMVEC apoptosis by administration of Ang–(1–7) in ACE2–deleted PMVECs exposed to LPS *in vitro*. In addition, whether Ang(1–7)/Mas receptor leads to the prevention of acute lung injury through MAPK/NF–kB signaling pathways *in vivo* should be addressed.

## Author Contributions

L.Y.C. proposed the hypothesis, designed the experiments and wrote the manuscript. C.Y.M. carried out the immunoassays. Z.Z. performed flow cytometry analysis and L.M.F. performed western–blot analysis. X.Y. and X.C.H. participated in the design of the study and performed the data analysis. Z.M. helped to edit the manuscript and J.W. conceived of the study, and participated in its design and coordination. All authors read and approved the final manuscript.

## Figures and Tables

**Figure 1:** Effects of ACE2 and Mas–receptor antagonist A779 on apoptosis of PMVECs treated with LPS for 48 h. (A) LPS exposure caused a significant apoptosis in PMVECs but was attenuated by ACE2 overexpression and aggravated by ACE2 downregulation. (B) LPS–induced apoptosis was markedly increased by A779 pretreatment but was improved by ACE2 overexpression. There was no significant difference between the ACE2 + A779 + LPS group and LPS group in apoptosis. All data are expressed as mean ± SD. * *P* < 0.05 compared with PBS control group; ^#^*P* < 0.05 compared with LPS group.

**Figure 2:** Effects of ACE2 and Mas–receptor antagonist A779 on cytokine secretion in PMVECs. (A, C) LPS exposure for 48 h caused a significant increase of the levels of IL–1β and TNF–α in the supernatants of cultured PMVECs but was markedly attenuated by ACE2 overexpression and aggravated by ACE2 downregulation. (B, D) LPS–induced IL–1β and TNF–α secretions were markedly increased by A779 pretreatment, but were improved by ACE2 overexpression. There was no significant difference in cytokine secretion between the ACE2 + A779 + LPS and LPS groups. All data are expressed as mean ± SD. * *P* < 0.05 compared with control group; ^#^*P* < 0.05 compared with LPS group.

The article "Angiotensin-converting enzyme 2/angiotensin-(1–7)/Mas axis prevents lipopolysaccharide–induced apoptosis of pulmonary microvascular endothelial cells by inhibiting JNK/NF–κB pathways" was retracted in 2026. Reasons: plagiarized images; duplicated images; overlap with other authors' work; overlap with earlier publications.

**Figure 3:** Effects of ACE2 and Mas–receptor antagonist A779 on AngII/Ang–(1–7) secretion in PMVECs. (A, C) LPS exposure for 48 h caused a significant increase of AngII and a slightly increase of Ang–(1–7). The increase of AngII was markedly attenuated by ACE2 overexpression and aggravated by ACE2 downregulation. The up–regulation of Ang–(1–7) was further increased by ACE2 overexpression, but reduced by ACE2 knockdown. (B, D) LPS–induced AngII secretion was markedly increased by A779 pretreatment, which was suppressed by ACE2 overexpression. But, Ang–(1–7) level was not affected by A779 pretreatment before LPS administration. All data are expressed as mean ± SD. * *P* < 0.05 compared with control group; ^#^*P* < 0.05 compared with LPS group.

**Figure 4:** Effects of ACE2 and Mas–receptor antagonist A779 on the ACE2/ACE expression in PMVECs. (A) LPS exposure for 48 h caused a significant decrease of the ACE2/ACE ratio in PMVECs that was markedly reversed by ACE2 overexpression and aggravated by ACE2 downregulation. (B) The ratio of ACE2/ACE was greatly reduced with A779 pretreatment prior to LPS stimulation that was reversed by ACE2 overexpression. There was no difference in the ACE2/ACE ratio between the A779 + LPS and LPS groups. All data are expressed as mean ± SD. * *P* < 0.05 compared with control group; ^#^*P* < 0.05 compared with LPS group.

**Figure 5:** Effects of ACE2 and Mas–receptor antagonist A779 on the phosphorylation of MAPKs in PMVECs. (A, C, E) LPS exposure for 48 h caused a significant increase in phosphorylation of ERK1/2, p38, and SAPK/JNK in PMVECs. ACE2 overexpression effectively reduced LPS–induced p38 and SAPK/JNK phosphorylation levels, but ERK1/2 phosphorylation was unaffected. In contrast, downregulation of ACE2 in LPS–exposed cells obviously enhanced ERK1/2 phosphorylation levels, but failed to change p38 and SAPK/JNK phosphorylation. (B, D, F) The phosphorylation levels of ERK1/2, p38, and SAPK/JNK were significantly enhanced by A779 pretreatment prior to LPS stimulation. ACE2 overexpression before A779 pretreatment obviously downregulated the levels of p38 and SAPK/JNK phosphorylation, but slightly decreased ERK1/2 phosphorylation level. All data are expressed as mean ± SD. * *P* < 0.05 compared with control group; ^#^*P* < 0.05 compared with LPS group; $ *P* < 0.05 compared with ACE2 + LPS group; ^&^*P* < 0.05 compared with A779 + LPS group.

**Figure 6:** Effects of ACE2 and Mas–receptor antagonist A779 on NF–κB p65 phosphorylation and IκBα expression in PMVECs. (A, B) LPS exposure for 48 h caused a significant increase in phosphorylation of NF–κB p65 and decrease in levels of IκBα in PMVECs. ACE2 overexpression effectively reduced LPS–induced NF–κB p65 phosphorylation levels and reversed IκBα levels. In contrast, downregulation of ACE2 in LPS–exposed cells obviously enhanced NF–κB p65 phosphorylation levels and suppressed IκBα levels. The phosphorylation of NF–κB p65 and downregulation of IκBα were significantly enhanced by A779 pretreatment prior to LPS stimulation. A779 pretreatment markedly reversed the effect of ACE2 overexpression on NF–κB p65 phosphorylation and IκBα expression. All data are expressed as mean ± SD. * *P* < 0.05 compared with the control group; ^#^*P* < 0.05 compared with the LPS group.

The article "Angiotensin-converting enzyme 2/angiotensin-(1–7)/Mas axis prevents lipopolysaccharide–induced apoptosis of pulmonary microvascular endothelial cells by inhibiting JNK/NF–κB pathways" was retracted in 2026. Reasons: plagiarized images; duplicated images; overlap with other authors' work; overlap with earlier publications.

**Figure 7:** Effects of the specific inhibitors of MAPKs on LPS–induced apoptosis in PMVECs. The protective effect of ACE2 overexpression on LPS–induced apoptosis was enhanced by SP600125 and deteriorated by SB203580 and PD98059. SP600125 markedly reduced apoptosis of PMVECs with *Ace2* deletion and Mas receptor blocker pretreatment. Mas receptor blocker abolished the protective effect of ACE2, which was aggravated by SB203580 and PD98059 and also SP600125. All data are expressed as mean ± SD. * *P* < 0.05 compared with PBS control group; ^#^*P* < 0.05 compared with LPS group; ^&^*P* < 0.05 compared with the ACE2 + LPS (A), shACE2 + LPS (B), A779 + LPS (C), and ACE2 + A779 + LPS (D) groups.

**Figure 8:** Effects of the specific inhibitors of MAPKs on LPS–induced cytokine secretion in PMVECs. (A, B) In the ACE2 + LPS group, SB203580, PD98059 and SP600125 pretreatment did not affect LPS–induced IL–1β and TNF–α secretions. (C, D) Pre–incubation with SB203580, PD98059, and especially SP600125, significantly suppressed the secretion of cytokines, in the shACE2 + LPS group. (E, F) In PMVECs exposed to LPS, pretreatment with A779 caused a significant increase in IL–1β and TNF–α secretions, which were slightly reduced by SB203580 and PD98059 as well as markedly attenuated by SP600125. (G, H) LPS–induced IL–1β and TNF–α secretions in the ACE2 + A779 + LPS group were significantly inhibited by SP600125 pre–incubation and were not affected by SB203580, or PD98059. All data are expressed as mean ± SD. * *P* < 0.05 compared with the PBS control group; ^#^*P* < 0.05 compared with the LPS group; ^&^*P* < 0.05 compared with the ACE2 + LPS (A), shACE2 + LPS (B), A779 + LPS (C), and ACE2 + A779 + LPS (D) groups.

## References

[b1] RubenfeldG. D. *et al.* Incidence and Outcomes of Acute Lung Injury. N Engl J Med 353, 1685–93 (2005).1623673910.1056/NEJMoa050333

[b2] PhuaJ. *et al.* Has mortality from acute respiratory distress syndrome decreased over time? : A systematic review. Am J Respir Crit Care Med 179, 220–7 (2009).1901115210.1164/rccm.200805-722OC

The article "Angiotensin-converting enzyme 2/angiotensin-(1–7)/Mas axis prevents lipopolysaccharide–induced apoptosis of pulmonary microvascular endothelial cells by inhibiting JNK/NF–κB pathways" was retracted in 2026. Reasons: plagiarized images; duplicated images; overlap with other authors' work; overlap with earlier publications.

[b3] ChengC. *et al.* Lipopolysaccharide induces expression of SSeCKS in rat lung microvascular endothelial cell. Mol Cell Biochem 305, 1–8 (2007).1755167010.1007/s11010-007-9521-7

[b4] WeirM. R. & DzauV. J. The renin–angiotensin–aldosterone system: a specific target for hypertension management. Am J Hypertens 12, 205S–213S (1999).1061957310.1016/s0895-7061(99)00103-x

[b5] de ManF. S. *et al.* Dysregulated renin–angiotensin–aldosterone system contributes to pulmonary arterial hypertension. Am J Respir Crit Care Med 186, 780–9 (2012).2285952510.1164/rccm.201203-0411OCPMC5104838

[b6] ChouC. H., ChuangL. Y., LuC. Y. & GuhG. Y. Interaction between TGF–beta and ACE2–Ang–(1–7)–Mas pathway in high glucose–cultured NRK–52E cells. Mol Cell Endocrinol 366, 21–30 (2013).2317475710.1016/j.mce.2012.11.004

[b7] SongB. *et al.* Loss of Angiotensin–Converting Enzyme 2 Exacerbates Myocardial Injury via Activation of the CTGF–Fractalkine Signaling Pathway. Circ J 77, 2997–3006 (2013).2416190610.1253/circj.cj-13-0805

[b8] TipnisS. R. *et al.* A human homolog of angiotensin–converting enzyme. Cloning and functional expression as a captopril–insensitive carboxypeptidase. J Biol Chem 275, 33238–43 (2000).1092449910.1074/jbc.M002615200

[b9] DonoghueM. *et al.* A novel angiotensin–converting enzyme–related carboxypeptidase (ACE2) converts angiotensin I to angiotensin 1–9. Circ Res 87, E1–9 (2000).1096904210.1161/01.res.87.5.e1

[b10] SantosR. A., FerreiraA. J., Verano–BragaT. & BaderM. Angiotensin–converting enzyme 2, angiotensin–(1–7) and Mas: new players of the renin–angiotensin system. J Endocrinol 216, R1–R17 (2013).2309287910.1530/JOE-12-0341

[b11] RiceG. I., ThomasD. A., GrantP. J., TurnerA. J. & HooperN. M. Evaluation of angiotensin–converting enzyme (ACE), its homologue ACE2 and neprilysin in angiotensin peptide metabolism. Biochem J 383, 45–51 (2004).1528367510.1042/BJ20040634PMC1134042

[b12] FerrarioC. M. & VaragicJ. The ANG–(1–7)/ACE2/mas axis in the regulation of nephron function. Am J Physiol Renal Physiol 298, F1297–305 (2010).2037511810.1152/ajprenal.00110.2010PMC2886811

[b13] JiaH. P. *et al.* ACE2 receptor expression and severe acute respiratory syndrome coronavirus infection depend on differentiation of human airway epithelia. J Virol 79, 14614–21 (2005).1628246110.1128/JVI.79.23.14614-14621.2005PMC1287568

[b14] ImaiY. *et al.* Angiotensin–converting enzyme 2 protects from severe acute lung failure. Nature 436, 112–6 (2005).1600107110.1038/nature03712PMC7094998

[b15] AsaduzzamanM., WangY. & ThorlaciusH. Critical role of p38 mitogen–activated protein kinase signaling in septic lung injury. Crit Care Med 36, 482–8 (2008).1809154610.1097/01.CCM.0B013E31816204FA

The article "Angiotensin-converting enzyme 2/angiotensin-(1–7)/Mas axis prevents lipopolysaccharide–induced apoptosis of pulmonary microvascular endothelial cells by inhibiting JNK/NF–κB pathways" was retracted in 2026. Reasons: plagiarized images; duplicated images; overlap with other authors' work; overlap with earlier publications.

[b16] SunS. X., GeB. X. & MiaoC. H. Effects of preconditioning with sevoflurane on TNF–alpha–induced permeability and activation of p38 MAPK in rat pulmonary microvascular endothelial cells. Cell Biochem Biophys 61, 123–9 (2011).2133658710.1007/s12013-011-9168-6

[b17] ZhouZ., ConnellM. C. & MacEwanD. J. TNFR1–induced NF–kappaB, but not ERK, p38MAPK or JNK activation, mediates TNF–induced ICAM–1 and VCAM–1 expression on endothelial cells. Cell Signal 19, 1238–48 (2007).1729258610.1016/j.cellsig.2006.12.013

[b18] GallagherP. E., FerratioC. M. & TallantE. A. MAP kinase/phosphatase pathway mediates the regulation of ACE2 by angiotensin peptides. Am J Physiol Cell Physiol 295, C1169–74 (2008).1876892610.1152/ajpcell.00145.2008PMC2585001

[b19] BrighamK. L. & MeyrickB. Endotoxin and lung injury. Am Rev Respir Dis 133, 913–27 (1986).3085564

[b20] FaffeD. S. *et al.* Respiratory effects of lipopolysaccharide–induced inflammatory lung injury in mice. Eur Respir J 15, 85–91 (2000).1067862610.1183/09031936.00.15108500

[b21] KaganJ. C. & MedzhitovR. Phosphoinositide–mediated adaptor recruitment controls Toll–like receptor signaling. Cell 125, 943–55 (2006).1675110310.1016/j.cell.2006.03.047

[b22] KawaiT. & AkiraS. Toll–like receptors and their crosstalk with other innate receptors in infection and immunity. Immunity 34, 637–50 (2011).2161643410.1016/j.immuni.2011.05.006

[b23] TogbeD. *et al.* Toll–like receptor and tumour necrosis factor dependent endotoxin–induced acute lung injury. Int J Exp Pathol 88, 387–91 (2007).1803927510.1111/j.1365-2613.2007.00566.xPMC2517336

[b24] ImaiY. *et al.* Identification of oxidative stress and Toll–like receptor 4 signaling as a key pathway of acute lung injury. Cell 133, 235–49 (2008).1842319610.1016/j.cell.2008.02.043PMC7112336

[b25] ShenW., GanJ., XuS., JiangG. & WuH. Penehyclidine hydrochloride attenuates LPS–induced acute lung injury involvement of NF–kappaB pathway. Pharmacol Res 60, 296–302 (2009).1938628210.1016/j.phrs.2009.04.007

[b26] ChoiM. S. *et al.* Inhibitory effect of obovatol on nitric oxide production and activation of NF–kappaB/MAP kinases in lipopolysaccharide–treated RAW 264.7cells. Eur J Pharmacol 556, 181–9 (2007).1713469310.1016/j.ejphar.2006.10.054

[b27] BadieiA., MunirajN., ChambersS. & BhatiaM. Inhibition of hydrogen sulfide production by gene silencing attenuates inflammatory activity by downregulation of NF–kappaB and MAP kinase activity in LPS–activated RAW 264.7 cells. Biomed Res 2014, 848570 (2014).10.1155/2014/848570PMC415186025215294

The article "Angiotensin-converting enzyme 2/angiotensin-(1–7)/Mas axis prevents lipopolysaccharide–induced apoptosis of pulmonary microvascular endothelial cells by inhibiting JNK/NF–κB pathways" was retracted in 2026. Reasons: plagiarized images; duplicated images; overlap with other authors' work; overlap with earlier publications.

[b28] LiuS., FengG., WangG. L. & LiuG. L. p38MAPK inhibition attenuates LPS–induced acute lung injury involvement of NF–kappaB pathway. Eur J Pharmacol 584, 159–65 (2008).1832847810.1016/j.ejphar.2008.02.009

[b29] FerreiraA. J. *et al.* Angiotensin–converting enzyme 2 activation protects against hypertension–induced cardiac fibrosis involving extracellular signal–regulated kinases. Exp Physiol 96, 287–94 (2011).2114862410.1113/expphysiol.2010.055277PMC3077555

[b30] SukumaranV. *et al.* Cardioprotective effects of telmisartan against heart failure in rats induced by experimental autoimmune myocarditis through the modulation of angiotensin–converting enzyme–2/angiotensin 1–7/mas receptor axis. Int J Biol Sci 7, 1077–92 (2011).2192757710.7150/ijbs.7.1077PMC3174385

[b31] ChenL. N. *et al.* Dysregulated renin–angiotensin system contributes to acute lung injury caused by hind–limb ischemia–reperfusion in mice. Shock 40, 420–9 (2013).2390385410.1097/SHK.0b013e3182a6953e

[b32] Wösten–van AsperenR. M. *et al.* Acute respiratory distress syndrome leads to reduced ratio of ACE/ACE2 activities and is prevented by angiotensin–(1–7) or an angiotensin II receptor antagonist. J Pathol 225, 618–27 (2011).2200955010.1002/path.2987

[b33] ZhongJ. *et al.* Angiotensin–converting enzyme 2 suppresses pathological hypertrophy, myocardial fibrosis, and cardiac dysfunction. Circulation 122, 717–28 (2010).2067954710.1161/CIRCULATIONAHA.110.955369

[b34] PhillipsM. I. & KagiyamaS. Angiotensin II as a pro–inflammatory mediator. Curr Opin Investig Drugs 3, 569–77 (2002).12090726

[b35] SuzukiY. *et al.* Inflammation and angiotensin II. Int J Biochem Cell Biol 35, 881–900 (2003).1267617410.1016/s1357-2725(02)00271-6

[b36] ZhangH. & SunG. Y. LPS induces permeability injury in lung microvascular endothelium via AT(1) receptor. Arch Biochem Biophys 441, 75–83 (2005).1609847310.1016/j.abb.2005.06.022

[b37] ShenoyV. *et al.* The angiotensin–converting enzyme 2/angiogenesis–(1–7)/Mas axis confers cardiopulmonary protection against lung fibrosis and pulmonary hypertension. Am J Respir Crit Care Med 182, 1065–72 (2010).2058117110.1164/rccm.200912-1840OCPMC2970847

[b38] KleinN. *et al.* Angiotensin–(1–7) protects from experimental acute lung injury. Crit Care Med 41, e334–43 (2013).2394947010.1097/CCM.0b013e31828a6688

[b39] SiddiquiS. S., SiddiquiZ. K., UddinS., MinshallR. D. & MalikA. B. p38 MAPK activation coupled to endocytosis is a determinant of endothelial monolayer integrity. Am J Physiol Lung Cell Mol Physiol 292, L114–L124 (2007).1689139010.1152/ajplung.00257.2005

[b40] LeeV. Y. *et al.* Bleomycin induces alveolar epithelial cell death through JNK–dependent activation of the mitochondrial death pathway. Am J Physiol Lung Cell Mol Physiol 289, L521–L528 (2005).1614805010.1152/ajplung.00340.2004

The article "Angiotensin-converting enzyme 2/angiotensin-(1–7)/Mas axis prevents lipopolysaccharide–induced apoptosis of pulmonary microvascular endothelial cells by inhibiting JNK/NF–κB pathways" was retracted in 2026. Reasons: plagiarized images; duplicated images; overlap with other authors' work; overlap with earlier publications.

[b41] UhalB. D., LiX., XueA., GaoX. & Abdul–HafezA. Regulation of alveolar epithelial cell survival by the ACE–2/angiotensin 1–7/Mas axis. Am J Physiol Lung Cell Mol Physiol 301, L269–74 (2011).2166596010.1152/ajplung.00222.2010PMC3174737

[b42] YunheF. *et al.* The effect of magnolol on the Toll–like receptor 4/nuclear factor kappaB signaling pathway in lipopolysaccharide–induced acute lung injury in mice. Eur J Pharmacol 689, 255–61 (2012).2268386410.1016/j.ejphar.2012.05.038

[b43] FanJ., YeR. D. & MalikA. B. Transcriptional mechanisms of acute lung injury. Am J Physiol Lung Cell Mol Physiol 281, L1037–50 (2001).1159789410.1152/ajplung.2001.281.5.L1037

[b44] AbrahamE. Nuclear factor–kappaB and its role in sepsis–associated organ failure. J Infect Dis 187, S364–9 (2003).1279285310.1086/374750

[b45] KarinM. & Ben–NeriahY. Phosphorylation meets ubiquitination: the control of NF–[kappa]B activity. Annu Rev Immunol 18, 621–63 (2000).1083707110.1146/annurev.immunol.18.1.621

[b46] BaeuerleP. A. & BaltimoreD. I kappa B: a specific inhibitor of the NF–kappa B transcription factor. Science 242, 540–6 (1988).314038010.1126/science.3140380

[b47] WangY. *et al.* Adenosine 5'–monophosphate–induced hypothermia inhibits the activation of ERK1/2, JNK, p38 and NF–kappaB in endotoxemic rats. Int Immunopharmacol 23, 205–210 (2014).2521816310.1016/j.intimp.2014.09.002

[b48] SchuhK. & PahlA. Inhibition of the MAP kinase ERK protects from lipopolysaccharide–induced lung injury. Biochem Pharmacol 77, 1827–34 (2009).1942833710.1016/j.bcp.2009.03.012

[b49] MengY. *et al.* Angiotensin–converting enzyme 2/angiotensin–(1–7)/Mas axis protects against lung fibrosis by inhibiting the MAPK/NF–kappaB pathway. Am J Respir Cell Mol Biol 50, 723–36 (2014).2416826010.1165/rcmb.2012-0451OC

